This article has been retracted.

# Luminal B tumors are the most frequent molecular subtype in breast cancer of North African women: an immunohistochemical profile study from Morocco

**DOI:** 10.1186/1746-1596-7-170

**Published:** 2012-12-07

**Authors:** Hinde El Fatemi, Sanae Chahbouni, Sofia Jayi, Kaoutar Moumna, My Abdelilah Melhouf, Abdelaziz Bannani, Omar Mesbahi, Afaf Amarti

**Affiliations:** 1 Department of Pathology, Hassan II teaching hospital, Fez, Morocco; 2 Department of Gynecology, Hassan II teaching hospital, Fez, Morocco; 3 Department of Oncology, Hassan II teaching hospital, Fez, Morocco

**Keywords:** Breast cancer, Molecular classification, Luminal B subtype, Staging, Antibodies, Immunohistochemistry

## Abstract

**Background:**

Breast cancer may be classified into luminal A, luminal B, HER2+/ER-, basal-like and normal-like subtypes based on gene expression profiling or immunohistochemical (IHC) characteristics. The aim of our study is to show the molecular profile characteristic of breast cancer in the North African population of Morocco. This work showed preliminary results and correlations with clinicopathological and histological parameters. Three hundred and ninety primary breast carcinomas tumor tissues were immunostained for ER, PR, HER2, CK5/6, CK8/18 and Ki67 using paraffin tissue.

**Methods:**

We reviewed 390 cases of breast cancer diagnosed on January 2008 to December 2011 at the Department of pathology, Hassan II teaching hospital, Fez, Morocco. Age, size tumor, metastatic profile, node involvement profile, histological type and immunohistochemical profile were studied.

**Results:**

The average age was 46 years; our patients were diagnosed late with a high average tumor size. Luminal B subtype was more prevalent (41.8%), followed by luminal A (30.5%), basal-like (13, 6%), Her2-overexpressing (9, 2%), and unclassified subtype (4.9%).

**Conclusion:**

This study showed that molecular classification and biological profile may be different according to geographical distribution, to encourage further studies to know the genomic profile of tumors and the environment.

**Virtual slide:**

http://www.diagnosticpathology.diagnomx.eu/vs/1675272504826544

## Background

Breast cancer is a heterogeneous disease such that they may have different prognoses and respond to therapy differently despite similarities in histological types, grade and stage. Based on the presence or absence of expression of the estrogen receptor (ER), breast cancer is divided in two groups: ER+ and ER-. Genetic expression profile has identified two subtypes of the ER+ tumors: luminal A and luminal B. ER- tumors also include two subtypes, the HER2+ and the basal type. These subtypes differ in their biology and both demonstrate short disease-free periods after treatment and poorer outcome. In Morocco, it’s the first cancer in women and is currently a major public health problem. The molecular classification in breast carcinomas is now based upon gene expression analysis using DNA microarrays and allows to identify at least five groups: luminal A, luminal B, HER2-overexpressing, basal-like and normal breast-like [1-3]. However, large-scale subtyping using gene expression profiling from formalin-fixed, paraffin-embedded samples is not currently feasible and remains very expensive. Therefore, immunohistochemical markers have been used as surrogates tools for DNA microarray in subtyping breast cancer [4,5]. Several studies used routinely panels of immunohistochemical markers to classify breast cancers into subtypes similar to those previously defined using gene expression analyses [6]. The recent study was realized by Prat et al. [4]. They defined several immunohistochemical subtypes: (luminal A, Luminal B, HER2- enriched, basal-like) and a normal breast-like group that show significant differences in incidence, survival and response to therapy. Luminal A (ER positive (ER+) and/or PR positive (PR+), Her2 negative (Her2-)) with ki67<14%, luminal B (ER + and/or PR+ with ki67>14%, Her2 positive or negative (Her2+/-), Her2+/ER − subtype (Her2+, ER−, PR−) and basal-like (ER−, PR−, Her2−, Cytokeratin 5/6 positive (CK5/6+) and/or Her1+ (EGFR)). Tumors which were negative at immunohistochemical staining for all markers (ER, PR, Her2, Her1, and CK5/6) were considered unclassified subtype [4]. According to this classification, we performed immunohistochemical staining for ER, PR, Her2, Her1, CK8/18, basal CK5/6 and KI67 in paraffin sections from blocks of breast cancer. The aim of the present study was to estimate the prevalence of breast cancer subtypes in patients of the north east region of Morocco, and to correlate between clinical and pathological characteristics.

## Methods

Patients this study was approved by Ethical Committee of Hassan II teaching hospital Center. A total of three hundred and ninety patients diagnosed with invasive breast carcinoma were examineted. Clinical information was retrieved from the medical records. Breast cancers were classified according to the World Health Organization (WHO, 2003) [7] while histological grading and staging were performed according to Modified Bloom-Richardson classification [8] and American Joint Committee on Cancer (AJCC) [9], respectively.

### Immunohistochemical study

Tumors sections were deparaffinized and rehydrated. Peroxide blocking was done with 0.4% H2O2. Antigen retrieval was achieved by heat retrieval using a pressure cooker. After washing, the slides were treated with protein blocking agent (UltraTech HRP, Immunotech) then incubated with the following primary antibodies: anti-human ER (ER1D5, Immunotech), PR (PR10A9, Immunotech), CK5/6 (D5/16B4, Cell Marque), CK8/18 (RTU-5D3, Novocastra), Ki67 (SP6 Cell Marque). After rinsing with PBS, the slides were incubated with a secondary biotinylated antibody (Immunotech). The slides were then rinsed with PBS. Sections were then incubated with streptavidin-peroxidase reagent. Staining for the slides was developed with Amino-Ethyl-Carbazole (Ultra Tech AEC, Immunotech) and then the slides were counterstained with hematoxylin, hydrated, and mounted. For Her2, immunohistochemical was carried out using with HercepTest (A0485, Dako) according to the commercial instructions for use.

Immunohistochemical surrogate biomarkers of molecular classification Immunohistochemical subtypes were defined as follows: Luminal A (ER + and/or PR+, Her2-, KI67<14%), luminal B (ER + and/or PR+, Her2+/-, Ki67>14%), basal-like (ER-, PR-, Her2-, and CK5/6+, CK14+), Her2+/ER-, and unclassified subtype (negative for all markers) (Table 1). CK8/18 expression was used for confirmation the luminal subtypes.

**Table 1:** Immunohistochemical characterization of molecular subtypes of breast cancer

**Molecular subtype**	**Immunohistochemical characterization**
Luminal A	ER (+) et Her-2 (-) et CK8/18 (+), Ki67<14%
Luminal B	ER (+) et Her-2 (+)
	ou ER (+), Her-2 (-) et Ki67>14%
Her-2	ER (-) et Her-2 (+)
Basal	ER (-) et Her-2 (-) et CK5/6 (+)

Positive controls were included in each staining run and consisted of breast cancers known to express each of the antigens of interest. Cases were considered positive for ER and PR according to standardized guidelines using a cut-off of ≥1% stained tumour nuclei. Fluorescence in situ hybridization (FISH) study

All Her2 score 2+ cases were analyzed by FISH. They were performed using the PathVysion HER2 DNA Probe (Abbott Vysis Inc., Downers Grove, IL) according to the manufacturer’s protocol. The probe cocktail included the LSI HER-2/neu probe and the CEP17 probe. Fluorescence signals were analyzed and digitalized using the CytoVisionTM image analysis system (Applied Imaging International Ltd., Newcastle-Upon-Tyne, UK). Between 60 and 100 nuclei were scored for each case. Signal ratios (HER2: CEP17) ≥ 2, 2 were classified as amplified. In the absence of positive FISH data, tumors scored 2+ by IHC were considered as negative for HER-2. Her2 was scored based on a 0 to 3 scale according to the criteria set by ASCO (American Society of Clinical Oncology/College of American Pathologists) [10]. Scores 0 and 1+ were considered as negative; score 2+ was considered borderline; and score 3+ was considered as strongly positive. FISH was performed on the borderline cases (score 2+).

### KI67

In breast cancer, immunohistochemical assessment of the proportion of cells staining for the nuclear antigen Ki67 has become the most widely used method for comparing proliferation between tumor samples. Potential uses include prognosis, prediction of relative responsiveness or resistance to chemotherapy or endocrine therapy, estimation of residual risk in patients on standard therapy and as a dynamic biomarker of treatment efficacy in samples taken before, during, and after neoadjuvant therapy, particularly neoadjuvant endocrine therapy. Cases were considered positive for ki67 according to standardized guidelines using a cut-off of ≥14% stained tumour nuclei with moderate intensity (Figure 1).

**Figure 1:** Distribution by the proliferation index assessed by Ki 67.

### Statistical analysis

Statistical analysis was performed in the Department of Epidemiology, of the Faculty of Medicine and Pharmacy of Fez and was carried out using Epi-Info (3.3.2).

## Results and discussion

The study was achieved on 390 patients diagnosed with infiltrating breast cancer and managed at the Department of pathology in Hassan II University Hospital in Fez. The patient’s average age at diagnosis was 46 years (ranging from 22 to 92 years). The tumor clinical stage on first diagnosis, according to American Joint Committee on Cancer Staging Systems, showed that 47 women (14.5%) are at stage I, 108 (33%) are at stage II, 114 (35%) are at stage III and 57 (17.5%) at stage IV. After histological analysis, the tumor average size was 3.7 ± 2.6 cm (ranging from 0.2 to 16 cm). Most of these tumors (87, 2%) were diagnosed as invasive carcinoma (IC NOS) while 5, 4% were invasive lobular carcinomas (ILC), 2% were metaplastic carcinoma (MC), and few patients had cancers of rare histology (5, 4%), which were summarized as “other types” in our study. The histological grade distribution for luminal B were grade II (59.9%), grade III (30.6%) but few patients only were grade I (9,6%) with p<0,0001. Vascular emboli were detected in 71.2% of patient’s luminal B. The status of lymph nodes was determined for 326 patients among which 68, 8% had positive lymph nodes and 12.5% had distant metastasis.

The immunohistochemical study showed that 67, 1% patients were ER positives, 63, 7% were PR positive, and 24, 7% were Her2 positive. Therefore, Luminal B subtype was more prevalent (41.8%), followed by luminal A (30.5%), basal-like (13, 6%), Her2-overexpressing (9, 2%), and unclassified subtype (4.9%). The luminal B subtypes present a higher median tumor size (T2 and T3) as like basal-like and Her2-overexpressing. IHC subtypes were significantly different by histological grade (p< 0.00001). The luminal B also represented a higher percentage of cases with histological grade II and III (90, 5%) like, basal-like and Her2-overexpressing subtypes (90, 2% and 96% respectively) and a very low percentage of tumors with histological grade I (9,6%, 9,8% and 4%, respectively). The Luminal B subtype had 71, 2% vascular emboli, approach Her2-overexpressing subtypes (75,6%). In this study, the luminal B tumors had average percentage of lymph node metastasis (68, 8%) and distant metastasis (12, 5%). Table 2 Twenty-two patients (12.2%) died because of cancer-related events during the follow-up. Among these patients, 25% belong to basal-like, 22% belong to unclassified subtype group. 20% to Her2-overexpressing group, 17% to luminal B and only 5% in luminal A.

**Table 2:** Prevalence of intrinsic subtypes and clinico-pathological characteristics

**subtype**	**luminal A**	**luminal B**	**Her-2**	**Basallike**	**Unclassified**
**Histological type %**					
**IDC Nos**	**30,5**	**41,1**	**10,9**	**13,9**	**3,6**
**ILC**	**47,6**	**42,9**	**4,8**	**0,0**	**4,8**
**Other types**	**25**	**8,3**	**16,7**	**50**	**0,0**
**P<0,00001**					
**Histological grade%**					
**I**	**28,3**	**9,6**	**9,8**	**4**	**15,8**
**II**	**59,2**	**59,9**	**56,1**	**32**	**26,3**
**III**	**12,5**	**30,6**	**34,1**	**64**	**57,9**
**P<0,0001**					
**Vascular emboli %**					
**Positive**	**60,8**	**71,2**	**75,6**	**64,4**	**63,2**
**negative**	**39,2**	**28,8**	**24,4**	**35,3**	**36,8**
**p=0,29**					
**Intraductal carcinoma %**					
**Yes**	**55**	**39,5**	**41,5**	**25,5**	**78,9**
**No**	**45**	**60,5**	**58,5**	**74,5**	**21,1**
**P=0,0013**					
**Tumour size (cm)**					
**T1**	**42,9**	**31,8**	**9,1**	**12,5**	**25**
**T2**	**34,5**	**44,76**	**45,5**	**46,9**	**25**
**T3**	**14,3**	**18,8**	**27,3**	**15,6**	**12,5**
**T4**	**8,4**	**4,7**	**18,2**	**25**	**37,5**
**P=0,0003**					
**Necrosis %**					
**Present**	**8,5**	**17,8**	**22,2**	**22,6**	**10,5**
**Absent**	**91,5**	**82,8**	**77,8**	**77,4**	**89,5**
**P=0,0698**					
**Positive Lymph nodes %**	**52,4**	**68,8**	**86,7**	**81,3**	**-**
**P=0,0066**					
**Distant metastasis %**					
**Yes**	**4,5**	**12,5**	**17,9**	**26,7**	**28,6**
**No**	**95,5**	**87,5**	**82,1**	**73,3**	**71,4**
**P=0,0030**					

Molecular studies of breast cancer revealed biological heterogeneity of the disease and opened new perspectives for personalized therapy. While multiple gene expression-based systems have been developed, current clinical practice is largely based upon conventional clinical and pathologic criteria. Digital image analysis (DA) with multivariate statistics of the data opens new opportunities in this field [11].

Recently, gene expression studies, using microarray technology, confirmed that the heterogeneity of clinical response could be correlated with different molecular profiles of breast cancers [1]. Arvydas and al reported a series of tissue microarrays of 109 patients with breast ductal carcinoma, were stained for a set of 10 IHC markers (ER, PR, HER2, Ki67, AR, BCL2, HIF-1α, SATB1, p53, and p16) [12]. This study demonstrates that factor analysis of multiple IHC biomarkers measured by automated DA is an efficient exploratory tool clarifying complex interdependencies in the breast ductal carcinoma IHC profiles. Major factor of the aggressive disease behaviour (i-Grade) is characterized by opposite loadings of ER/PR/AR/BCL2 and Ki67/HIF-1α. The i-Grade factor scores represent integral quantitative characteristics that reveal bimodal distribution and are strongly associated with the histological grade and relevant intrinsic subtypes. In HR-positive tumours, the aggressiveness of the tumour is best reflected by the combination of Ki67 and ER, rather than Ki67 and BCL2. Inverse relation between HER2 and PR expression in the HR-positive tumours which, along with the inverse relation between Ki67 and ER, may shed the light into the differential information conveyed by the ER and PR expression. Remarkably, SATB1 along with HIF-1α reflected the second major factor of variation in patients with breast cancer; furthermore, in the HR-positive group they were inversely associated with the HR and BCL2 expression and represented the major factor contributing to the variation in the IHC data set. However, this factor was not associated with the clinicopathologic categories studied. Biological meaning of this variation remains unclear: HIF-1α and SATB1 may convey important biological messages other than the aggressiveness of the disease reflected by Ki67 expression and histological grade. Meanwhile, the authors, support the notion that the suggested prognostic significance of SATB1 may be related to its inverse relation to the ER expression. Finally, this analysis confirms high expression levels of p16 in Triple-negative tumours [12]. In our study, based on recent updated IHC subtype definition by Prat et al. [4], we estimated the prevalence of breast cancer subtypes in patients from the north east Moroccan region and established the correlations between clinico-pathological characteristics. The patients recruited in our university hospital were younger than in western series; the average age at diagnosis was 46.8 years. In terms of clinical staging, only 14.5% patients were diagnosed at stage I, while 33% were at stage II, 35% at stage III and 17.5% at stage IV. On the other hand, after histological analysis the average tumor size was 3.7 cm and 75% of cases measured more than 2 cm. A majority of tumors were stage II or III. Our data showed that more than 50% of patients of all subtypes presented positive lymph nodes and more than 12% of cases had distant metastasis on first diagnosis. This could be due to late consultation during the progression of the disease in our region as well as to lack of the Medicare coverage, lack of screening mammography program and women’s awareness trainings particularly in rural area. The predominant histology type in this study was invasive cancer (87.4%), similar to most breast cancer studies worldwide. Overexpression of the protein and/or amplification of the HER2 gene have been reported in approximately 20 to 30% of breast cancers, similar to what was found in our patients (24,7%). Her2+ tumors are associated with either poor prognosis or with response to trastuzumab [13]. Our results showed a distribution of breast cancer subtypes non similar to what was reported by other immunohistochemical studies [4]. In this study, the prevalence of luminal B (41, 8%) and is the more frequent subtype. Considering the fact that all patients came from a university hospital the possible effects of a selection bias should be regarded. Cancer registry available includes only data from the university hospital and not all North African population of Morocco. Triple-negative subtype represented approximately 13, 6% of our series and 78% of them were basal-like tumors. These results were similar to what was found in other studies [4,14]. The basal-like group was defined by immunohistochemistry, as being negative for ER, PR, and Her2 and positive for Ck5/6, CK14 and/or Her1 (EGFR). It is important to study whether EGFR is overexpressed in patients with breast cancer since these patients can be given specific EGFR molecule tyrosine kinase inhibitors such as gefitinib and lapatinib [15,16]. There are only a few reports regarding the overexpression of EGFR, with these studies indicating 8-36% of breast cancers over express this protein. However, systematic studies appraising EGFR gene amplification and mutations in the same set of cases among Chinese female patients with breast cancer are absent [17-19]. EGFR gene mutations are infrequent in breast cancers. This suggested that EGFR mutation analysis is not useful as a screening test for sensitivity to anti-EGFR therapy for breast cancers [20]. In literature, the luminal B tumors are associated with poor recurrence-free and disease-specific survivals in all adjuvant systemic treatment categories including hormone therapy; the identification of specific signaling pathways driving luminal B biology is paramount to improve treatment. Sircoulomb et al. and Holland et al. have independently identified the ZNF703 gene, located in chromosomal region 8p12, as preferentially amplified in luminal B tumours [21].

The natural history of breast cancer involves progression through defined pathological and clinical stages, starting with ductal hyperproliferation, with subsequent evolution into in situ and invasive carcinomas, and finally into metastatic disease. The majority of invasive breast cancer develop over long periods of time from certain pre-existing benign lesions. The best characterized premalignant lesions recognized today are referred to as atypical ductal hyperplasia (ADH), atypical lobular hyperplasia (ALH), ductal carcinoma in situ (DCIS) and lobular carcinoma in situ (LCIS). Douglas and al, [22] reported that Lobular neoplasia (LN) and invasive lobular carcinoma (ILC) are detected together frequently in the same specimen and location of the tumor--in up to 90% of cases of ILC [23]. Invasive carcinomas were present with LN in 45.6% of cases, with similar rates of association with invasive carcinoma and ILC (47.2%). Bratthauer and Tavassoli stratified the LNs as "lobular intraepithelial neoplasias" (LIN) and evaluated the frequency of association between LIN subtypes (1, 2, and 3) and invasive carcinoma. The percentage of LIN 1 (equivalent to ALH) that was associated with invasive carcinoma was 14%, and 89% of these tumors were IDCs. In the patients with LIN 3 (equivalent to LCIS), the frequency of association with IDC and ILC was 23% and 86%, respectively. The authors concluded that the advance from LIN 1 to LIN 3 was linked to a 64% increase in the frequency of invasive carcinoma and a greater than 70% rise in the likelihood of ILC [24]. Apoptosis is a frequent phenomenon in breast cancer and it can be detected by light microscopy in conventional histopathological sections or by special staining techniques. Balance between expression status of anti-apoptotic and pro-apoptotic proteins determines cells to be alive or not. The key event of apoptosis occurrence is cascade activation of caspases, and inhibitor of apoptosis proteins (IAPs) play a important role in caspase inhibition. XIAP is the most potent caspase inhibitor and Smac is one of the antagonists of XIAP. Down regulation of XIAP expression or applying exogenous Smac mimics can sensitize tumor cells, especially for breast cancer cells, to chemotherapeutics and promote apoptosis [25,26]. In immunohistochemistry, XIAP and Smac were positive in cytoplasm of tumor cells with strong or moderate intensity, respectively. The positive ratio of XIAP (84.3%, 86/102) was more higher than that of Smac (33.3%, 34/102), and immunoscore of XIAP was higher than Smac in IDC too (*P* < 0.0001). It was noteworthy that 44 IDC samples were nuclear positive for XIAP, but none was for Smac. And cytoplasm positive status of XIAP nuclear positive group was stronger than the negative group (*P* = 0.030, 0.047). Otherwise, Smac immunoscore was prevalent in HER2 positive group than negative group (*P* < 0.0001). Remaining data revealed that the expression status of XIAP/Smac was not correlated with patient age, tumor size, lymph node status, histologic grading, expression of ER and PR. XIAP was a potent protein for apoptosis inhibition and Smac was an important negative regulator of the former. Disturbed balance of expression between XIAP and Smac probably contributed to carcinogenesis and XIAP positive nuclear labeling was a sign of unfavourable prognosis in breast invasive ductal carcinoma [27]. Others studies have demonstrated that claudin-6 functions as a cancer suppressor in human MCF-7 breast cancer cells. The growth inhibitory effect could be attributed to inhibition of cell proliferation and induction of apoptosis. Claudins (CLDNs) constitute a family of integral membrane proteins and have been identified as prominent structural components of tight junction ( TJ ) strands [28,29]. TJs are junctional complexes which mediate cell-to-cell adhesion in epithelial and endothelial cellular sheets [30], and which affect cell polarity and tight junction formation [28]. Guo and al reported that the apoptosis signal-regulating kinase 1 (ASK1) expression is low in breast cancer, and the levels of ASK1 mRNA and protein expression are correlated with that of claudin-6. They have identified a novel mechanism responsible for the pro-apoptosis function of claudin-6, and ASK1 may become a target for breast cancer treatments. The integrins, a family of transmembrane glycoproteins, play a major role in invasive and metastatic processes. Integrins are involved in cell adhesion in both cell-extracellular matrix and cell-cell interactions, and particularly, beta 1 integrin is involved in proliferation and differentiation of cells in the development of epithelial tissues. The putative role of beta 1 integrin expression on survival and metastasis in patients with breast invasive ductal carcinoma (IDC) was studied by Santos and al [31]. His study showed that beta1 integrin can be a marker of poor prognosis in breast cancer. Beta 1 integrin was overexpressed in 32.8% of IDC and was related with HER-2 and VEGF expression, and it had a significant relationship with metastasis and death , survival analysis showed that the overexpression of this protein is very significant in specific survival (number of months between diagnosis and death caused by the disease). Immunohistochemistrey is important to determinate the tumors of unknown origin (5-15%) and specially breast cancer metastasis (1.5%). Mammaglobin (MAG) antibody in the immunohistochemical panel for the detection of tumors of unknown origin contributed to the detection of metastasis of breast cancer. The diagnostic strategy with the highest positive predictive value (88%) included hormone receptors and mammaglobin in serial manner [32].

## Conclusions

We have shown that simple IHC-based classification of breast tumors can be helpful. Since the predictive power of IHC criteria appears to be similar to that of gene expression analysis, this information can be used to improve therapeutic decisions, mainly for luminal B, Her2- overexpressing and basal-like subtypes. The luminal B subtype was associated with a poor prognosis and unfavorable clinico-pathological characteristics. In addition, findings concerning tumors stages are alarming and highlight the importance of early screening and the urgent need to improve women’s awareness of breast cancer in our region. Our results should be confirmed by large studies to be conducted in other institutions and hospitals including patients coming from different regions of Morocco.

## Abbreviations

HER2: Epithelial human receptor 2; ER: Estrogen receptor; PR: Progesterone receptor; IHC: Immunohistochemistry; CK: Cytokeratin; WHO: World Health Organization; AJCC: American Joint Committee on Cancer; FISH: Fluorescence in situ hybridization; IC NOS: Invasive carcinoma not otherwise specified; ILC: Invasive lobular carcinoma; MC: Metaplastic carcinoma; DA: Digital image analysis; EGFR: Epidermal growth factor receptor; ADH: Atypical ductal hyperplasia; ALH: Atypical lobular hyperplasia; DCIS: Ductal carcinoma in situ; LCIS: Lobular carcinoma in situ; LN: Lobular neoplasia; LIN: Lobular intraepithelial neoplasia; ASK1: Apoptosis signal-regulating kinase 1.

## Competing interests

The authors declare that they have no competing interests.

## Authors’ contributions

All authors analyzed, interpreted and approved the final manuscript.

## Funding

This study received no specific grant from any funding agency in the public, commercial or not-for-profit sectors
